# Effects of Scrambler Therapy in Patients with Failed Back Surgery Syndromes and Factors Associated with Depression Affecting Pain before and after the Therapy

**DOI:** 10.1155/2020/9342865

**Published:** 2020-07-05

**Authors:** Hayoung Byun, Min-Kyun Oh, Chang Han Lee

**Affiliations:** Department of Rehabilitation Medicine, Gyeongsang National University, School of Medicine, Gyeongsang National University Hospital, Jinju, Republic of Korea

## Abstract

**Objectives:**

To report the effects of scrambler therapy in patients diagnosed with failed back surgery syndromes and to analyze the factors affecting pain before and after the therapy.

**Methods:**

This study included 26 patients (12 males and 14 females). The Oswestry Disability Index (ODI) and Brief Pain Inventory (BPI) before and after scrambler therapy, Beck Depression Inventory (BDI) score before therapy, and residual pain after therapy were assessed. The changes in the ODI, BPI, and residual pain before and after the therapy were analyzed using the Wilcoxon signed rank test. Spearman correlation analysis and Fisher's exact test were used to confirm the correlation between BDI and other factors. Multiple regression analysis was used to identify independent factors predicting residual pain, posttherapy ODI, and posttherapy BPI.

**Results:**

The ODI changed from 25.69 ± 7.98 to 21.80 ± 9.41 (*p* < 0.05), and the BPI changed from 68.96 ± 18.00 to 61.62 ± 20.27 after scrambler therapy (*p* < 0.05). In addition, residual pain changed from 100 to 76.15 (*p* < 0.05). The BDI was negatively correlated with the duration of scrambler therapy and positively correlated with the initial OPD and BPI. In multiple regression analysis, residual pain was significantly correlated with the BDI (*p* < 0.05).

**Conclusion:**

Scrambler therapy can be used to change the total scores of the ODI and BPI after 5 sessions of treatment. Also, residual pain was significantly related to the BDI. Clinical significance of depression severity on pain should be further investigated via prospective studies.

## 1. Introduction

The overall incidence of low back pain is estimated at 9.4%, which is a global challenge causing more disability than any other disease [1]. In addition to suffering and disability, low back pain has a considerable impact on society. Due to the significant increase in the prevalence of back pain over time, it is plausible that the rate of surgery for the treatment of back pain has continued to increase similarly [2]. Occasionally, however, surgery may not relieve patient's pain or may provide only a temporary relief. Failed back surgery syndrome represents a constellation of conditions that describe persistent or recurring low back pain, with or without sciatica following one or more spine surgeries [3].

The treatment of failed back surgery syndrome is similar to that of chronic back pain, and the options range from conservative treatment to invasive procedures such as epidural injection and ultimately to surgery. In general, revision surgeries are not associated with improved pain score and involve a high rate of complications such as increased bleeding, infections, and acute respiratory distress syndrome [4]. Therefore, appropriate selection of treatment considering the cause of pain, and based on the success and risk of the procedure, is required in patients with failed back surgery syndrome [5].

Scrambler therapy is an effective conservative treatment used to treat patients with failed back surgery syndrome without side effects [6]. Giuseppe Marineo who developed scrambler therapy reported that chronic pain is one of the typical neuropathies resulting from persistent pain delivery [7]. He claimed that the loss of the cause-effect linear relationship in acute pain may contribute to a novel, nonlinear relationship with chronic pain in the pain system. Therefore, intervention at the level of afferent pain mechanism may be used to control chronic pain [7].

Depression is closely related to not only acute but also chronic pain. Gilles et al. [8] found that the presence of postoperative acute pain was related to anxiety and depression. Carr et al. [9] also suggested that depression scores increased following the increased pain after gynecological surgery. The prevalence of pain symptom was 51.8–59.1% in patients with depression [10, 11], and the prevalence of depression was 13–85% in patients with chronic pain [12]. In addition, depressive symptoms were among the predictors of neck and low back pain [13]. Therefore, depression might alter the treatment efficacy of chronic pain and vice versa.

This study was aimed to report the effects of scrambler therapy in patients with failed back surgery syndrome. It also analyzed the factors that affect pain before and after scrambler therapy.

## 2. Materials and Methods

### 2.1. Study Design and Participant Selection

This was a pre-post comparison study conducted in the Department of Rehabilitation Medicine at a university hospital. The study was approved by the Institutional Review Board of our Hospital. It was conducted from November 2018 to July 2019.

Individuals with persistent back pain after surgical interventions for spine were investigated when scrambler therapy was selected as the treatment option. The inclusion criteria were as follows: (i) subjects aged between 30 and 70 years and (ii) preliminary diagnosis of failed back surgery syndrome. Subjects were excluded under one of the following conditions: (i) acute myocardial infarction or ischemic heart diseases for the last six months; (ii) pregnancy or lactation; (iii) hypersensitivity to transcutaneous nerve stimulator or allergy to rubber; (iv) mesentery nerve block or neuropathy treatment for the last four weeks; (v) severe arrhythmia or abnormality on electrocardiogram; (vi) wound or skin disorder associated with the painful back; and (vii) poor compliance.

### 2.2. Standardized Scrambler Therapy

Pain Jammer (ENS-1140, Korea) was used for scrambler therapy. Each scrambler therapy consisted of a 50-min daily session for 5 consecutive days, Monday through Friday. For the therapy, the most symptomatic area of low back and buttock region was determined based on patient report. Electrodes were placed around and along the lines of pain and numbness. After appropriate positioning of the electrode pairs, the device was turned on, and the patient was told that the electrode intensity would be raised to the maximally tolerated intensity. The stimulation intensity increased until the patient felt a sting or burning sensation. The researcher informed that sensory stimulation would change to a tingling sensation. When the sensory stimulus was still a sting, burn, or induced discomfort after increasing stimulation intensity, electrodes were moved laterally further than before, and the therapy was restarted with zero intensity. During the therapy, the patient was informed that the stimulation intensity would increase to the maximally tolerated intensity without any discomfort. When the stimulation was too strong, the researcher decreased the intensity without eliciting patient discomfort. When the patient notified maximum stimulation intensity of tolerance, any preexisting pain was evaluated. After the pain disappeared, the aforementioned procedures were repeated around the painful area to treat residual pain.

### 2.3. Outcome Measurements

Informed consent was obtained from all patients, and demographics such as age, height, weight, and gender were collected at the time of enrollment. The patients also were asked to complete the pain and depression questionnaires.

#### 2.3.1. Pain Outcome Measurements

Outcome measurements were performed before and one week after the therapy. The degree of physical disability, pain status, and the degree of pain relief after the therapy were measured.

The degree of physical disability was measured using the Oswestry Disability Index (ODI) [14]. The patients were asked to complete a questionnaire containing six statements (denoted levels 0–5) in each of the 10 sections related to impairment: pain, personal care, lifting, walking, sitting, standing, sleeping, sex life, social life, and traveling. In each section, the patient was asked to select the statement that best described his/her status. The total score ranged from 0 (highest level of function) to 50 (lowest level of function). To accommodate patients who failed to respond to every section, the percentage of disability was calculated depending on the total number of possible points.

The severity of pain was evaluated using the Brief Pain Inventory (BPI) questionnaire. The BPI is composed of pain severity score and pain interference score [15]. The BPI pain severity score includes 4 items scored with numeric rating scales based on patients' subjective rating of their pain intensity on a 0–10 point scale. Each scale is presented as a row of equidistant numbers where 0 = no pain and 10 = worst possible pain. The patient's functional status was measured according to the 7 items using the BPI pain interference score measured on a scale of 0–10, with 0 denoting “no interference” and 10 suggesting “interference completely” with regard to the extent of pain interference with enjoyment of each item. Lastly, residual pain after the therapy compared with the baseline was determined based on patient's subjective evaluation of improvement after the therapy considering the maximum intensity of pain before the therapy as 100%. For example, if the patient stated that his/her pain after the therapy was half of the pain before the therapy, the residual pain was recorded as 50%.

#### 2.3.2. Depression Measurement

The Beck Depressive Inventory (BDI) was used to assess depression in patients with failed back surgery syndrome. The BDI is a widely used tool to evaluate the presence and severity of depression. It is a multiple choice self-administered inventory consisting of 21 items. Each item is evaluated on a scale ranging from 1 to 3 (three corresponds to the most severe) [16]. The BDI scores between 0 and 13 indicate minimal depression; from 14 to 19 indicate mild depression; 20 to 28 indicate moderate depression; and 29 to 63 indicate severe depression.

### 2.4. Statistical Analysis

The Wilcoxon signed rank test was used to compare the total score of the ODI, BPI, and residual pain before and after scrambler therapy. Spearman correlation analysis and Fisher's exact test were used to confirm the correlation between the BDI and other factors. Since the results of the BDI score were continuous variants, we divided the BDI score into four groups: minimal (0–13), mild (14–19), moderate (20–28), and severe categories (29–63). Multiple regression analysis and multinomial logistic regression analysis were used to identify independent factors predicting residual pain, posttherapy ODI, and posttherapy BPI. The assessed data were analyzed using the Statistical Package for Social Science for Windows ver. 20.0 (SPSS Inc., Armonk, NY, USA), and the level of significance was set at *p* < 0.05.

## 3. Results

### 3.1. General Characteristics of Subjects

Twenty-six patients diagnosed with failed back surgery syndrome were enrolled after meeting our inclusion criteria. All subjects completed the study in accordance with the study protocol, and no subjects reported complications or issues associated with the use of pain scrambler therapy. General characteristics of the subjects are listed in Table 1.

### 3.2. Changes in Total ODI and BPI Scores

The mean initial ODI total score was 25.69 ± 7.98, and the ODI score 1 week after the therapy was 21.80 ± 9.41. The mean initial BPI total score was 68.96 ± 18.00, and the BPI total score 1 week after the therapy was 61.62 ± 20.27. There were significant changes in the total ODI and BPI scores at 1 week after the therapy compared with the baseline (Table 2). The mean residual pain was 76.15 ± 4.21 after the therapy, which was significantly different compared with the baseline value (Table 2).

### 3.3. Relationship between Various Factors and BDI

Age, height, weight, BMI, gender, and type of surgery were not correlated with the BDI (*p* > 0.05), but there was a significant negative correlation between duration of scrambler therapy and the BDI (*r* = −0.422, *p*=0.032). In addition, significant positive correlation was found between the BDI and initial levels of the ODI and BPI (Table 3).

### 3.4. Factors Affecting Residual Pain, Posttherapy ODI, and Posttherapy BPI

In multiple regression analysis where the residual pain was a dependent variable, the initial ODI, initial BPI, age, and BMI were not significantly correlated, whereas the BDI was correlated with residual pain (Table 4). Also, multinomial logistic regression analysis showed that gender was not significantly related to the residual pain (Table 4).

Multiple regression analysis and multinomial logistic regression analysis of posttherapy ODI revealed the effects of residual pain (*p*=0.127), initial ODI (*p*=0.000), initial BPI (*p*=0.152), age (*p*=0.667), BMI (*p*=0.145), BDI (*p*=0.144), and gender (*p*=0.176) (Table 5). Also, multiple regression analysis and multinomial logistic regression analysis of posttherapy BPI revealed the effects of residual pain (*p*=0.000), initial ODI (*p*=0.207), initial BPI (*p*=0.000, age (*p*=0.111), BMI (*p*=0.481), BDI (*p*=0.761), and gender (*p*=0.695) (Table 5). Thus, the initial ODI was significantly correlated with posttherapy ODI, and initial BPI was significantly correlated with posttherapy BPI.

## 4. Discussion

In this study, scrambler therapy reduced the pain scores measured by the ODI and BPI after one week treatment. It also decreased the residual pain. Depression score was negatively correlated with the duration of scrambler therapy and positively correlated with the initial pain scores measured by the ODI and BPI. In addition, the residual pain was significantly correlated with the depression score.

The primary aim of this study was to compare the pain scores before and after scrambler therapy, and the study showed changes in the pain scores after 1 week of treatment. Scrambler therapy is a new instrument designed to replace “pain” information with the “nonpain” information via noninvasive cutaneous electric stimulation. This instrument generates 16 different currents that stimulate normal nerve action potentials similar to endogenous nerve action potentials and consists of an algorithm based on output, frequency, duration, amplitude modulation, and other factors. The stimulus was delivered via cutaneous electrodes around the painful area, and the pain was decreased if the electrodes were placed appropriately. The information is processed via replacement of intrinsic pain information with “nonpain” or “normal” information through the C-fiber surface receptor, which may be delivered to the brain. The plasticity of brain networks that induces pain perception allows the replacement of “pain” information with “nonpain” information [17]. In the double-blinded, randomized controlled trial of 30 subjects with lower back pain, scrambler therapy showed a significant decrease in the “worst” pain and interference scores, and the findings correlated with our results [6].

Transcutaneous electrical nerve stimulation (TENS) also has been used to treat postoperative and musculoskeletal pain. It is known to reduce pain via central and peripheral mechanisms. It centrally activates the spinal cord and brainstem where the opioid, serotonin, and muscarinic receptors are activated [18]. However, limited randomized controlled trials investigated the effects of TENS on neuropathic pain [18]. In contrast, scrambler therapy has revealed its effects on neuropathic pain. The pilot trial involving 11 cancer patients who had abdominal pain showed that scrambler therapy significantly reduced pain from 8.6 to 2.3 after 10 sessions [7]. In the study of 16 patients with refractory chemotherapy-induced neuropathic pain, pain scores were reduced by 58% after 10 sessions of scrambler therapy [19]. In the randomized controlled trial of Marineo et al. [17], scrambler therapy relieved chronic neuropathic pain better than drugs based on treatment guidelines.

The mechanism of pain modulation by scrambler therapy has yet to be elucidated, and further studies are needed. However, this study is consistent with previous studies investigating scrambler therapy. First, scrambler therapy delivers “nonpain” information at the pain area [17]. Using five channels of electrical stimulation in scrambler therapy, the surface receptors of C-fibers replace endogenous pain information with a synthetic “nonpain” or “normal-self” information that travels along the same pathways to the brain. Based on this plasticity within the brain networks mediating pain perception, a series of treatments “retrain” the brain, so that the area of concern is no longer considered painful. If this “nonpain” information is eliminated, scrambler therapy is merely an electrical stimulation, which is not effective in pain relief and instead produces pain [20]. Patients in this study also showed relevant pain relief after the standard protocol of scrambler therapy, when the pain information was replaced with tolerable painless information such as tingling sensation. Since the standard protocol was based on the replacement of pain with “nonpain” information, no patient failure or side effects were detected. This study electrically stimulated patients for 50 min, which may be sufficient to allow the delivery of pain messages by the surface receptors of C-fibers to the pain perception area of the brain. Therefore, the study results support the theory of Marineo, who developed scrambler therapy [20].

Second, the pain relief effects were sustained for days, which may suggest either resetting of calcium channels or remodulation of the pain response [17]. Patients in this study, similar to others treated with scrambler therapy, experienced pain relief lasting for at least one week after the therapy. Although the precise mechanism is unknown, the duration of the sustained effect may explain possible alteration at the cellular or biomolecular level.

The second aim of this study was to analyze the factors affecting pain before and after scrambler therapy. The study showed similar relationship between pain and depression score. Depression is known to be more common in patients with chronic pain than in healthy controls [21]. In addition, it is one of the strongest predictors for low back pain [22]. Based on the cross-sectional and cohort study comprising over 50,000 subjects reported by Meyer et al., depression and low back pain were correlated with a correlation coefficient of about 0.4, and the associational odds ratios increased with the intensity of back pain and severity of depression [23].

This study also showed a significant relationship between depression severity and pain severity before and after the therapy. Pain and depression are related to each other via biological pathways. First, depletion of serotonin and norepinephrine may interrupt the pain modulation in the rostral ventromedial medulla and dorsolateral pontine tegmentum, as in depression. This loss of modulation amplifies minor signals regarded as pain, which is not regarded as pain under normal circumstances [24]. A few experimental studies have shown that treatment with intrathecal serotonin and norepinephrine blocks pain signals [25, 26], and antidepressants that increase the levels of serotonin and norepinephrine affect pain modulation [27]. Second, brain regions associated with emotion, such as medial prefrontal, insular and anterior temporal cortex, hypothalamus, and amygdala, transmit signals to brainstem structures involved in pain modulation. Studies have shown that negative expectation about stimuli activates anterior cingulate cortex, parietal operculum, and posterior insula and exacerbates pain severity, while distraction from the stimuli decreases the activation and pain perception [28]. Therefore, the positive relationship between initial pain severities and the depression score in this study, as well as the significant relationship between the depression score and the residual pain may explain the biological validity of scrambler therapy similar to other pharmacological and nonpharmacological strategies for reducing pain. Unlike residual pain, multiple regression analysis of ODI and BPI scores after therapy were not significantly related to BDI. The initial ODI was the only significant predictor of posttherapy ODI, and the initial BPI was the only significant predictor of posttherapy BPI probably because the ODI and BPI assessments contain other components in addition to pain, such as social life and functional status [14, 15]. The significant relationship between residual pain and BDI, but not ODI and BPI, may suggest that residual pain rather than ODI or BPI explains the changes in pain.

The negative relationship between treatment duration and BDI can be explained by the nonstatic phenomenon of chronic pain. Bendayan et al. [29] found that depression slightly but constantly decreased eventually in patients with acute and chronic back pain. Also, the longitudinal study of depression in patients with spinal cord injury revealed that the prevalence of a probable major depression changed from 22.1% to 20.2% over time [30]. Adjustment to the injury and pain symptoms might lead to the highest depression score at the time of injury, which then decreases with time [31, 32]. The study result suggests the importance of depression treatment in patients with chronic pain such as failed back surgery syndrome, along with pain control treatment. No subject in this study was under depression treatment, which suggests underestimation of depression in patients with chronic pain. Therefore, increased consideration of depression or depressive symptoms when treating chronic pain patients may lead to better prognosis.

This study had limitations associated with small sample size of 26 subjects and lack of control (placebo or sham). A long-term follow-up may be needed to determine the long-term effects of scrambler therapy.

This study demonstrates that scrambler therapy may significantly reduce pain, which may be influenced by depression. Further investigation of scrambler therapy using long-term follow-up studies is essential to develop treatment and awareness about pain and depression. Also, further studies investigating brain networks might facilitate the exploration of the role of cerebral plasticity in pain perception.

## Figures and Tables

**Table 1:** Characteristics of subjects.

Characteristics	Value
Age (years)	67.8 ± 9.98
Gender	
Male	12
Female	14
Height (cm)	160.2 ± 11.65
Weight (kg)	63.0 ± 8.57
Body mass index (kg/m^*2*^)	24.68 ± 3.24
BDI	
Minimal	8
Mild	3
Moderate	5
Severe	10
Types of back surgery (multiple choice)	
Laminectomy	8
Discetomy	7
Posterior fusion	5
Anterior fusion	1
Posterolateral fixation	8
Vertebroplasty	1
Partial corpectomy	1
Treatment duration (months)	68.46 ± 9.33

Values are presented as mean ± standard deviation or number.

**Table 2:** Changes in the total ODI and BPI scores.

	Initial	1 week after the therapy	*p* value
ODI	25.69 ± 7.98	21.80 ± 9.41	0.000^a^
BPI	68.96 ± 18.00	61.62 ± 20.27	0.000^a^
Residual pain	100	76.15 ± 4.21	0.000^a^

Values are presented as mean ± standard deviation. ODI, Oswestry Disability Index; BPI, Brief Pain Inventory. ^a^*p* < 0.05, comparing initial scores with scores a week after therapy via the Wilcoxon signed rank test.

**Table 3:** Correlation between BDI and other factors.

	*r*	*p* value
Age	0.210	0.303^a^
Height	−0.052	0.800^a^
Weight	−0.219	0.281^a^
BMI	−0.223	0.273^a^
Treatment duration	−0.422	0.032^ac^
Initial ODI	0.796	0.000^ac^
Initial BPI	0.744	0.000^ac^
Gender		0.730^b^
Type of surgery		1.430^b^

ODI, Oswestry Disability Index; BPI, Brief Pain Inventory; BDI, Beck Depression Inventory. ^a^Spearman correlation analysis, ^b^Fisher's exact test, ^c^*p* < 0.05.

**Table 4:** Association between residual pain and various factors.

	*β*	*p* value
Initial ODI	−0.081	0.733
Initial BPI	−0.008	0.973
Age	−0.061	0.697
BMI	0.055	0.694
BDI	0.867	0.000^a^
Gender	0.255	0.383

*β*, standardized coefficient; ODI, Oswestry Disability Index; BPI, Brief Pain Inventory; BMI, body mass index; BDI, Beck Depression Inventory. ^a^*p* < 0.05.

**Table 5:** Association between various factors associated with posttherapy ODI and BPI.

	Posttherapy ODI		Posttherapy BPI	
	*β*	*p* value	*β*	*p* value
Initial ODI	0.755	0.000^a^	0.050	0.207
Initial BPI	0.296	0.152	0.838	0.000^a^
Age	−0.063	0.667	−0.040	0.111
BMI	−0.197	0.145	−0.019	0.481
BDI	0.296	0.144	−0.012	0.761
Gender	0.235	0.176	0.154	0.695

*β*, standardized coefficient; ODI, Oswestry Disability Index; BPI, Brief Pain Inventory; BMI, body mass index; BDI, Beck Depression Inventory. ^a^*p* < 0.05.

## Data Availability

The data used to support the findings of this study are available from the corresponding author upon request.
